The article "Up-regulation of miR-130b expression level and down-regulation of miR-218 serve as potential biomarker in the early detection of human osteosarcoma" was retracted in 2016. Reasons: misconduct by an author; plagiarized text; compromised peer review; false authorship.

# Up-regulation of miR-130b expression level and down-regulation of miR-218 serve as potential biomarker in the early detection of human osteosarcoma

**DOI:** 10.1186/s13000-015-0422-x

**Published:** 2015-10-07

**Authors:** Afshin Taheriazam, Amir Jouya Talaei, Mohammad Jamshidi, Mohammadreza Shakeri, Samaneh Khoshbakht, Emad Yahaghi, Marjan Shokrani

**Affiliations:** Department of Orthopedics Surgery, Tehran Medical Sciences Branch, Islamic Azad University, Tehran, Iran; Department of Genetics, Faculty of Life Sciences, Azad University of Tehran Medical Sciences Branch, Tehran, Iran; Cellular and Molecular Research Center, Zahedan University of Medical Sciences, Zahedan, Iran; Department of Clinical Biochemistry, School of Medicine, Zahedan University of Medical Sciences, Zahedan, Iran; Department of Orthopaedic and Trauma Surgery, Birjand University of Medical Sciences, Birjand, Iran; Department of Statistics, Faculty of Sciences, Islamic Azad University, Mashhad Branch, Mashhad, Iran; Department of Molecular Biology, Baqiyatallah University of Medical Sciences, Tehran, Iran; Graduate, Faculty of Medicine, Tehran University of Medical Sciences, Tehran, Iran

**Keywords:** Mir-130b/218, Osteosarcoma, Regulation, Patient, Diagnosis

## Abstract

**Background:**

Osteosarcoma (OS) is a primary malignant bone tumor with high morbidity that principally emerges in children and adolescents. MiRNAs regulate a variety of normal physiologic processes and are involved in tumorigenesis and development of multiple malignancies, including OS. This study was aimed to evaluate the clinical significance of miR-130b and miR-218 in osteosarcoma patient.

**Methods:**

We utilized quantitative real-time PCR to evaluate the level of miR-130b and miR-218 expressions in OS patients and normal tissues and their relationship with clinicopathological features and survival in OS patients.

**Results:**

QRT-PCR indicated that miR-130b expression in tumor tissues was strongly elevated than adjacent non-tumor tissues (*P* < 0.001), while the level of miR-218 expression in osteosarcoma tissues was down-regulated than adjacent non-tumor tissues (*P* < 0.001). We evaluated the clinical significance of miR-130b and miR-218 in osteosarcoma. Clinical correlation analysis showed that increased expression of miR-130b and decreased expression of miR-218 were significantly associated with advanced tumor stage (*x*^2^ = 6.285, *P* < 0.009; *x*^2^ = 7.172, *P* < 0.007), distant metastasis (*x*^2^ *= 5.528; P* < 0.001; *x*^2^ = 4.617, *P* < 0.001) and size of tumor (*x*^2^ = 5.01, *P* = 0.013; *x*^2^ = 4.271, *P* = 0.019).

**Conclusions:**

Taken together, our data indicated that high miR-130b level and low level of miR-218 are associated with poor clinicopathological characteristics. Furthermore, miR-130b may play a key role in the progression of osteosarcoma.

The article "Up-regulation of miR-130b expression level and down-regulation of miR-218 serve as potential biomarker in the early detection of human osteosarcoma" was retracted in 2016. Reasons: misconduct by an author; plagiarized text; compromised peer review; false authorship.

## Background

Osteosarcoma (OS) is a primary malignant bone tumor with high morbidity in children and young adults; hat is more common in males than in females [1–4]. Despite current treatments combining chemotherapy, surgery, the 5-year cumulative survival rate of primary osteosarcoma was only 50 %–60 % [5, 6]. Therefore, the discovery of new biomarkers for the diagnosis, prognosis, and treatment of OS remains an important but unmet clinical need. miRNAs are a family of small, non-coding, endogenous RNAs, that inhibit gene expression by binding to the 3′untranslated region (3′-UTR) of mRNA sequence, leading to translational degradation or repression [7, 8]. Studies have also shown that miRNAs are involved in tumor genesis and cancer progression. MiRNAs can function as either tumor suppressors or oncogenes according to their target genes [9, 10]. Many miRNAs are deregulated in various cancer subtypes [11–14].

MiRNAs have been indicated to be correlated with the proliferation, differentiation, apoptosis and invasion of tumor cells [15]. However, the role of miRNAs in osteosarcoma development has only recently been investigated and further investigations are needed to clarify the role miRNAS in terms of osteosarcoma. MiR-130b has been studied in various types of human cancers [16–20]. Down-regulation of miR-130b has been reported in endometrial cancer, pituitary adenomas, papillary thyroid carcinoma, and pancreatic cancer [18–21]. Nevertheless, it has been shown that miR-130b expression was aberrantly increased in melanoma, colorectal cancer, bladder cancer, and gastric carcinoma [16, 17, 22–24].

MiR-218 has been reported to be significantly deregulated in many kinds of tumors [25–30]. It was down-regulated in lung, prostate, cervical, colon, gastric, bladder cancer and hepatocellular carcinoma [25–29]. Moreover, decreased expression of miR-218 was related to a significant worse survival of HCC patients. Down regulation of miR-218 was found in osteosarcoma tissues [31]. Moreover, it has been reported that miR-218 inhibited osteosarcoma cell migration and invasion by down-regulating T-cell lymphoma invasion and metastasis 1 (TIAM1), matrix metalloproteinase2 (MMP2) and MMP9 [31]. However, it is important to evaluate the clinical significance of miR-130b and miR-218 in osteosarcoma patients.

## Materials and methods

Ethical approval for the study was obtained according to the Declaration of Helsinki. All subjects were volunteers and informed consents were obtained.

### Patients and tissue specimens

Cancerous tissues and adjacent non-tumor tissues (>3 cm distance to the resection margin) were obtained from 30 patients who underwent curative resection of osteosarcoma between December 2007 and September 2013 in Mashhad and Tabriz hospitals, Iran. All clinical samples were used after obtaining informed consent. Moreover, histological subtype and tumor grade were determined using the World Health Organization (WHO) criteria (Fig. 1). The tissues were stored at −80 °C until use. Union for International Cancer Control (UICC) tumor-nodemetastases (TNM) Staging Classification was used for the staging of the tumor. The clinical features of all enrolled patients were shown in Table 1.

The article "Up-regulation of miR-130b expression level and down-regulation of miR-218 serve as potential biomarker in the early detection of human osteosarcoma" was retracted in 2016. Reasons: misconduct by an author; plagiarized text; compromised peer review; false authorship.

**Fig. 1:** Expression levels of miR-130b and miR-218 in osteosarcoma tissues and adjacent non-tumor tissues

### RNA extraction and qRT-PCR

Briefly, total RNA was extracted from the tissues using TRIzol reagent (Invitrogen, Carlsbad, CA, USA), according to the manufacturer’s instructions. Two microliters of cDNA obtained from each sample was amplified and quantified by real-time PCR of TaqMan Human MiRNA Assay (Applied Biosystems) according to the manufacturer’s protocol. MiRNAs expressions relative to U6 were evaluated using the comparative cycle threshold (CT) method.

**Table 1:** Association between the clinicopathological parameters and expression of miRNAs in the osteosarcoma patients

Clinicopathological features	No. of cases	Expression of miR-130b		Expression of miR-218		*P* value of miR-130b	*P* value of miR-218
		Low = 11	High = 19	Low = 17	High = 13		
Gender						0.741	0.712
Male	17	7	10	11	6		
Female	13	4	9	6	7		
Age						0.517	0.483
<24	12	4	8	7	5		
≥25	18	7	11	10	8		
Tumor diameter (cm)						0.013	0.019
≤6	16	9	7	6	10		
>6	14	2	12	11	3		
Histology						0.51	0.503
Conventional osteosarcoma	20	6	14	11	9		
Others	10	5	5	6	4		
Clinical stage						0.009	0.007
I	12	8	4	4	8		
II	10	3	7	6	4		
III	8	0	8	7	1		
Distant metastasis						<0.001	<0.001
No	18	8	10	7	11		
Yes	12	3	9	10	2		

### Statistical analysis

The GraphPad Prism 5 software (GraphPad Software, Inc., San Diego, CA, USA) was applied for chi-square test and Two-tailed Student’s *t* test. Differences were considered statistically significant when *p* was less than 0.05.

## Results and Discussion

QRT-PCR indicated that miR-130b expression in tumor tissues was strongly elevated than adjacent non-tumor tissues (1.04 ± 0.31 vs. 0.59 ± 0.12, *P* < 0.001; Fig. 2), while the level of miR-218 expression in osteosarcoma tissues was down-regulated than adjacent non-tumor tissues (0.61 ± 0.21 vs. 1.53 ± 0.42, *P* < 0.001; Fig. 2).

**Fig. 2:** Pathology of osteosarcomas. High-powered photomicrographs of human osteosarcoma*s* show condensation of the neoplastic cells (H&E)

We evaluated the clinical significance of miR-130b and miR-218 in osteosarcoma. Clinical correlation analysis showed that increased expression of miR-130b and decreased expression of miR-218 were significantly associated with advanced tumor stage (*x*^2^ = 6.285, *P* < 0.007; *x*^2^ = 7.172, *P* < 0.009), distant metastasis (*x*^2^ *= 5.528; P* < 0.001; *x*^2^ = 4.617, *P* < 0.001) and size of tumor (*x*^2^ = 5.01, *P* = 0.013; *x*^2^ = 4.271, *P* = 0.019), (Table 1).

The article "Up-regulation of miR-130b expression level and down-regulation of miR-218 serve as potential biomarker in the early detection of human osteosarcoma" was retracted in 2016. Reasons: misconduct by an author; plagiarized text; compromised peer review; false authorship.

These results suggested that high miR-130b level and low level of miR-218 are associated with poor clinicopathological characteristics.

There is growing evidence that miRNAs can act as either oncogenes or tumor suppressor, depending on their target genes. Dysregulation of miRNAs has been linked to different malignancies [32, 33]. It has been already reported that different kinds of miRNAs are up-regulated or underexpressed in OS tissues and cell lines. These miRNAs are involved in occurrence and development of many kinds of tumors [34]. Down-regulation of miR-130b has been documented in endometrial cancer, pituitary adenomas, papillary thyroid carcinoma, and pancreatic cancer [18–21]. On the other hand, it was shown that miR-130b expression was increased in melanoma, colorectal cancer, bladder cancer, and gastric carcinoma [16, 17, 22–24]. Our findings indicated that miR-130b expression was strongly elevated in tumor tissues when compared with adjacent non-tumor tissues. Clinical correlation analysis showed that increased expression of miR-130b was significantly associated with advanced tumor stage, distant metastasis and size of tumor. These results suggested that high miR-130b level is associated with poor clinicopathological characteristics. Elevated expression level of miR-130b was associated with poorer prognosis of osteosarcoma patients. A previous study indicated that in CRC miR-130b induces EMT through a pathway that appears to be independent of DICER1 and its downstream target miR-200c. Moreover, the PPARγ is as a direct functional target of miR-130b in colorectal cancer. PPARγ is a CRC-independent prognostic factor implicated in cell differentiation and suppression of cell growth likely through up-regulation of its target genes E-cadherin, p21, and PTEN in colorectal cancer [17]. It has been found that, miR-130b could contribute to EMT of cancer cells by targeting DICER1 [35]. The involvement of miR-130b in CRC-related angiogenesis and EMT has been previously shown. In hypoxic conditions, miR-130b represses DDX6 leading to increased activity of HIF1α, a well-known VEGF inducer.

Furthermore, deregulation of miR-218 was reported in many kinds of tumors [25–30]. Down-regulation of it has been found in lung, prostate, cervical, colon, gastric, bladder cancer and hepatocellular carcinoma [25–29]. Moreover, decreased expression of miR-218 was related to a significant worse survival of HCC patients. Down regulation of miR-218 was found in osteosarcoma tissues [31]. Moreover, it has been reported that miR-218 inhibited osteosarcoma cell migration and invasion by down-regulating T-cell lymphoma invasion and metastasis 1 (TIAM1), matrix metalloproteinase2 (MMP2) and MMP9 [31]. In the present study, the level of miR-218 expression in osteosarcoma tissues was down-regulated in comparison with adjacent non-tumor tissues. We evaluated the clinical significance of miR-218 in osteosarcoma. Clinical correlation analysis showed that decreased expression of miR-218 was significantly associated with advanced tumor stage, distant metastasis and size of tumor. These results suggested that low level of miR-218 is associated with poor clinicopathological characteristics.

The article "Up-regulation of miR-130b expression level and down-regulation of miR-218 serve as potential biomarker in the early detection of human osteosarcoma" was retracted in 2016. Reasons: misconduct by an author; plagiarized text; compromised peer review; false authorship.

It has been reported that the low level of miR-218 is associated with TNM stage, lymph node metastasis and histological differentiation in colon cancer. Moreover, patients with low miR-218 expression had shorter survival in colon cancer [27]. Lower level of miR-218 has been found in patients with large tumor size and advanced TNM tumor stage in hepatocellular carcinoma tissues [30]. Our findings suggested that that miR-218 may be a potential marker in osteosarcoma patients. A previous study indicated that LEF1 is a new direct target of miR-218, and miR-218 can reduce protein levels of LEF1 and MMP-9 in glioblastoma cells. They hypothesized that miR-218 can directly target LEF1, resulting in reduced synthesis of MMP-9. Moreover, they concluded that miR-218 is involved in the invasive behavior of GBM cells and by targeting LEF1 and blocking the invasive axis, miR-218-LEF1-MMPs, it may be useful for developing potential clinical strategies [36]. Jin et al. [31] indicated that miR-218 can act as inhibitor of osteosarcoma cell migration and invasion by down-regulating TIAM1, MMP2 and MMP9 expression [18]. However, further studies are needed to clarify the role of miR-218 in osteosarcoma cell proliferation and apoptosis.

## Conclusions

In summary, our data indicated that high miR-130b level and low level of miR-218 are associated with poor clinicopathological characteristics. Furthermore, miR-130b may play a key role in the progression of osteosarcoma.

## Abbreviations

OS: Osteosarcoma
3′-UTR: 3′untranslated region
CT: Cycle threshold
UICC: Union for International Cancer Control
WHO: World Health Organization
TNM: Tumor-nodemetastases
TIAM1: T-cell lymphoma invasion and metastasis1
MMP2: Matrix metalloproteinase2
